RETRACTED

# High Expression of PTGR1 Promotes NSCLC Cell Growth via Positive Regulation of Cyclin-Dependent Protein Kinase Complex

**DOI:** 10.1155/2016/5230642

**Published:** 2016-06-26

**Authors:** Xianping Huang, Weihe Zhou, Yuefeng Zhang, Yong Liu

**Affiliations:** Department of Cardiothoracic Surgery, The Second Affiliated Hospital of Wenzhou Medical University, Wenzhou, Zhejiang 325027, China

## Abstract

Lung cancer has been the most common cancer and the main cause of cancer-related deaths worldwide for several decades. PTGR1 (prostaglandin reductase 1), as a bifunctional enzyme, has been involved in the occurrence and progression of cancer. However, its impact on human lung cancer is rarely reported. In this study, we found that PTGR1 was overexpressed in lung cancer based on the analyses of Oncomine. Moreover, lentivirus-mediated shRNA knockdown of PTGR1 reduced cell viability in human lung carcinoma cells 95D and A549 by MTT and colony formation assay. PTGR1 depletion led to G2/M phase cell cycle arrest and increased the proportion of apoptotic cells in 95D cells by flow cytometry. Furthermore, silencing PTGR1 in 95D cells resulted in decreased levels of cyclin-dependent protein kinase complex (CDK1, CDK2, cyclin A2, and cyclin B1) by western blotting and then PTGR1 is positively correlated with cyclin-dependent protein by using the data mining of the Oncomine database. Therefore, our findings suggest that PTGR1 may play a role in lung carcinogenesis through regulating cell proliferation and is a potential new therapeutic strategy for lung cancer.

## 1. Introduction

Lung cancer is still one of the major public health problems and the main risk factor of cancer-related deaths worldwide. There were an estimated 1.825 million new cases (12.9% of the total cancers), with nearly one death out of every five cases (1.59 million deaths, 19.4% of the total) in 2012 [1, 2]. In China, there were 652,842 new lung cancer cases and 597,182 deaths in 2012 according to GLOBOCAN 2012 data. Notably high incidence was observed in adult men who smoked [3]. Lung cancer is classified into two main histologic subtypes: small cell lung cancer (SCLC) and non-small cell lung cancer (NSCLC) which is the most common type accounting for 85% of all lung cancer cases. Because most NSCLC tumors develop slowly, they are generally diagnosed in the late stages with malignant proliferation and distant metastasis [4]. Thus, the novel and noninvasive prognostic biomarkers for treatment of NSCLC are extremely needed.

Human PTGR1 (prostaglandin reductase 1) gene is also named ZADH3 (zinc binding alcohol dehydrogenase domain containing 3) and LTB4DH (leukotriene B4 12-hydroxydehydrogenase), which was first cloned and identified from kidney cDNA libraries by Yokomizo et al. [5]. PTGR1 gene encodes a protein named LTB4DH or 15-oxoprostaglandin 13-reductase, which is a dual-functional enzyme capable of catalyzing the oxidation of LTB4 and the reduction of 15-oxo-prostaglandins (15-PGs) and 15-oxo-lipoxin A4 [6, 7]. PTGR1 has been shown to be involved in the regulation of inflammation via controlling the expression levels of specific eicosanoids in mycobacterial infection under physiological condition [8]. The substrates/products of PTGR1 in tumors are unbalanced and this imbalance can promote tumor growth. The expression levels of PTGR1 were increased during hepatocellular carcinoma (HCC) development in a time-dependent manner [9]. Tapak et al. reported that overexpression of PTGR1 was associated with a decrease in survival time in bladder cancer [10]. Additionally, the levels of PTGR in patients developing oral mucositis were significantly higher than in those not developing oral mucositis [11]. However, the biological function of the PTGR1 gene in NSCLC is scarce.

RETRACTED

In the current study, we explored the expression of PTGR1 in human NSCLC by using Oncomine database. We further investigated the function and preliminary mechanism of PTGR1 on the proliferation and apoptosis of NSCLC cells by using lentivirus-mediated interference of PTGR1 expression. What is more, the action of PTGR1 during tumorigenesis may provide the evidence to point at this enzyme as a possible therapeutic target for NSCLC.

## 2. Materials and Methods

### 2.1. Oncomine Analysis

The expression level of PTGR1 genes in NSCLC was analyzed using Oncomine (https://www.oncomine.org/) [12]. To this end, we compared clinical specimens of NSCLC versus normal tissues in four separate datasets (Beer Lung [13], Okayama Lung [14], Garber Lung [15], and Hou Lung [16]). Also, we extracted the mRNA expression value of PTGR1 and cyclin-dependent protein in the same samples of Hou Lung dataset to make the correlation analysis. For lowering the false discovery rate, we selected *p* < 0.05 as a threshold. The results were analyzed by their *p* values and cancer subtype. The log-transformed and normalized expression values of PTGR1 were extracted, analyzed, and read from the scatterplot.

### 2.2. Human Tissues and Cell Lines Culture

Ten pairs of human lung cancer tissues and corresponding normal tissues were obtained from the Department of Cardiothoracic Surgery, the Second Affiliated Hospital of Wenzhou Medical University, for the qRT-PCR assay. This research was authorized by the Ethics Committee of the Second Affiliated Hospital of Wenzhou Medical University, and informed consent form was obtained from each subject in accordance with the Helsinki Declaration. Human NSCLC cell lines, 95D cells (Cat. number TCHu61), A549 cells (Cat. number TCHu150), and human embryonic kidney 293T cells (HEK293T, Cat. number GNHu17), were obtained from the Cell Bank of the Chinese Academy of Sciences (Shanghai, China). 95D cells were cultured in Roswell Park Memorial Institute 1640 medium (RPMI 1640, Hyclone, SH30809.01B+) containing 10% fetal bovine serum (FBS, Biowest, Cat. number S1810). Both 293T and A549 cells were routinely cultured in Dulbecco's Modified Eagle's Medium (DMEM, Hyclone, Cat. number SH30243.01B+) supplemented with 10% FBS at 37°C in a 90% humidity incubator containing 5% CO_2_.

RETRACTED

### 2.3. shRNA Interference Vector Construction and Infection

PTGR1 (NCBI accession number NM_001146108) shRNA sequence was 5′- GCCTACTTTGGCCTACTTGAACTCGAGTTCAAGTAGGCCAAAGTAGGCTTTTT-3′ and control (no target for any genes) shRNA sequence was 5′-GCGGAGGGTTTGAAAGAATATCTCGAGATATTCTTTCAAACCCTCCGCTTTTTT-3′. Two stem-loop-stem sequences corresponding oligos were annealed and inserted into the linearized pFH-L vector (Shanghai Hollybio, China) which was digested by* NheI* and* PacI*. The related products were transformed into the competent cells of* E. coli* strain DH5*α* and purified by the Plasmid Mini Kit (Qiagen, Cat. number 12125). The lentiviral based shRNA-expressing vectors were determined by DNA sequencing. Lentivirus particle which could encode shPTGR1 or shCon was generated by cotransfection of HEK293T cells with packaging plasmids pVSVG-I and pCMVΔR8.92 (Shanghai Hollybio, China) using CaPO_4_ precipitation according to published protocols as previously described [17]. The supernatants were collected after 48 h. The pooled supernatants were centrifuged and filtered through a 0.45 *μ*m filter to remove cell debris and then concentrated by ultracentrifugation for 90 min at 83,000 g. The viral titer was measured by end point dilution analysis through counting the numbers of infected green fluorescence protein- (GFP-) positive cells under a fluorescence microscope (100x magnification, Olympus, Tokyo, Japan). Titer in IU/mL is calculated as follows: (the numbers of green fluorescent cells) × (dilution factor)/(volume of virus solution) [18]. 95D (100,000 cells/well) and A549 (30,000 cells/well) lung cancer cells were seeded in 6-well plates, respectively, and transfected with the constructed lentivirus containing shPTGR1 or shCon at a multiplicity of infection (MOI) of 60 and 50, respectively. Infection efficiency was determined and the efficiency of endogenous PTGR1 silencing was measured via quantitative real-time PCR (qRT-PCR) and western blot analysis.

RETRACTED

### 2.4. RNA Extraction and Real-Time PCR Analysis

The total RNA was collected from 95D and A549 cells after 5 and 8 days of lentivirus infection, respectively, by using TRIzol® reagent (Life Technologies, Cat. number 15596-018). The first-strand complementary DNA (cDNA) was synthesized using M-MLV reverse transcriptase (Promega, Cat. number M1705) in a total volume of 20 *μ*L reaction system containing 2 *μ*g total RNA. The PCR reaction mixtures contained 10 *μ*L of iQ*™* SYBR® Green Supermix (Bio-Rad, Cat. number 1708882AP), 0.5 *μ*M primers, and 0.8 *μ*L of cDNA. The CFX96 Touch*™* Real-Time PCR Detection System (Bio-Rad) was used to run qRT-PCR reaction. The primer sets were as follows: *β*-actin, 5′-GTGGACATCCGCAAAGAC-3′ (forward) and 5′-AAAGGGTGTAACGCAACTA-3′ (reverse), and PTGR1, 5′-TCCTCCTGTGACCCTTTCGG-3′ (forward) and 5′-GAAGGCGGCTGGGACTGC-3′ (reverse). The PCR reaction mixture was run as follows: initial denaturation at 95°C for 1 min, 40 cycles of denaturation at 95°C for 5 s, and extension at 60°C for 20 s. The relative gene expression level was calculated using the 2^−ΔΔCT^ method with normalization to the internal control *β*-actin.

### 2.5. Protein Extraction and Western Blotting

After 7 days and 6 days of the recombinant lentivirus shCon or shPTGR1 infection in 95D and A549 cells, respectively, cells were homogenized in ice-cold 2x sodium dodecyl sulfate (SDS) sample buffer (100 mM Tris-HCl (pH 6.8), 10 mM EDTA, 4% SDS, and 10% glycine). The concentration of total protein was analyzed using a BCA Protein Assay Kit (Pierce Biotechnology, Cat. number 23235). The protein samples (30 *μ*g/well) were separated by 10% SDS-polyacrylamide gel electrophoresis (PAGE) and electrotransferred to polyvinylidene difluoride (PVDF) membranes. The membranes were blocked in the sealing solution at room temperature for 1 h. Then, the membranes were incubated with rabbit anti-PTGR1 (Abgent, Cat. number BP5941c, 1 : 1,000 dilution), rabbit anti-CDK1 (Proteintech, Cat. number 19532-1-AP, 1 : 1000 dilution), rabbit anti-CDK2 (Cell Signaling Technology, Cat. number #2546, 1 : 1000 dilution), rabbit anti-cyclin A2 (Proteintech, Cat. number 18202-1-AP, 1 : 1000 dilution), rabbit anti-cyclin B1 (SAB, Cat. number #21540, 1 : 1000 dilution), and rabbit anti-GAPDH (Proteintech, Cat. number 10494-1-AP, 1 : 40,000 dilution) overnight at 4°C. After washing with TBST (TBS with 0.1% Tween 20) three times, incubation was carried out with goat anti-rabbit HRP secondary antibody (Santa Cruz, Cat. number SC-2054, 1 : 5,000 dilution) for 1 h at room temperature. Signals were detected using the ECL-PLUS/Kit (Amersham, Cat. number RPN2132) following the manufacturer's protocol. GAPDH was used as an internal control.

RETRACTED

### 2.6. MTT Assay

After lentivirus infection for 96 h and 72 h separately, lung cancer cells 95D and A549 were inoculated in 96-well plates at 3000 cells/well and 2000 cells/well, respectively. From the first day, MTT (3-(4,5-dimethylthiazol-2-yl)-2,5-diphenyltetrazolium bromide) was used to evaluate the rate of cell proliferation once daily for 5 days. Then, 20 *μ*L of MTT (Sigma, 5 mg/mL) was added to each well. After incubation for 4 h, the reaction was terminated by dimethyl sulfoxide (DMSO) at a volume of 100 *μ*L per well and then the plate was shocked at low speeds in a shaker for 10 min to dissolve the formazan thoroughly. The optical density (OD) value at 595 nm was measured using the Epoch Microplate Spectrophotometer (Biotek, CA, USA).

### 2.7. Colony Formation Assay

Colony formation assay was carried out according to previous report [19]. Briefly, lung cancer cells 95D and A549 (500 cells/well) were recultured in 6-well plates and continuously incubated for 8 days and 10 days, respectively. Then, the cell colonies were washed with PBS, fixed by 4% paraformaldehyde for 30 min, and stained with crystal violet (Beyotime, Cat. number C0121) for 10 min. The single colony with more than 50 cells was imaged and counted under light/fluorescent microscopy. Image analysis was conducted using Metamorph version 7.5 software (Molecular Devices, CA, USA).

### 2.8. Flow Cytometric Cell Cycle Analysis

Propidium iodide (PI) staining was applied to the analysis of cell cycle distribution through flow cytometry as previously described [20]. Briefly, approximately 80,000 cells were recultured in 6 cm dishes after lentivirus infection for 4 days in 95D cells. Subsequently, the cells were collected after 3 days, fixed in 70% prechilled ethanol overnight at 4°C, washed with prechilled PBS, and handled with 300 *μ*L staining solution containing 50 *μ*g/mL PI and 50 *μ*g/mL RNase A in the dark for 30 min in turn. Then, the DNA content was measured via FACSCalibur flow cytometer (Becton Dickinson, CA, USA). Data were analyzed with the ModFit DNA analysis program.

### 2.9. Annexin V-APC/7-AAD Staining Apoptosis Analysis

To examine apoptotic cells, the Annexin V-APC/7-AAD Apoptosis Detection Kit (KeyGen Biotech, Cat. number KGA1026) was used. 95D cells were seeded in 6 cm dishes at 80,000 cells/dish after 7 days of lentivirus infection, with additional culture of 40 h, and cells were harvested and stained as per the manufacturer's instructions. The cells were analyzed on FACSCalibur (Beckman Coulter, CA, USA) using CellQuest Pro software. The percentage of each quadrant was calculated.

### 2.10. Statistical Analysis

GraphPad Prism 5.0 software (GraphPad Software Inc., La Jolla, CA, USA) was applied to the data analysis. The data were analyzed using Student's *t*-test and expressed as mean ± SD. Pearson's correlation coefficient was determined between PTGR1 and cyclin-dependent protein expressions of NSCLC using GraphPad Prism 5.0 software. Values of *p* < 0.05 were considered statistically significant.

RETRACTED

## 3. Results

### 3.1. PTGR1 Is Highly Expressed in NSCLC Tissues

The relative expression levels of PTGR1 gene in NSCLC were systematically assessed by inquiring the Oncomine database. We compared PTGR1 expression in cancer versus normal tissues and in different cancer subtypes. PTGR1 differential expression analysis in NSCLC versus normal tissues showed 4 dataset results which showed a significant difference value of gene expression (*p* ≤ 0.05) in Oncomine database. PTGR1 expression is significantly elevated in lung adenocarcinoma (ADC, *n* = 86, *p* = 0.003) tumors compared to normal lung tissues (*n* = 10, Figure 1(a)) in Beer et al.'s study. Also, PTGR1 is overexpressed in ADC tumors (*n* = 226, *p* = 1.27*E* − 7) against normal tissues (*n* = 20, Figure 1(b)) in Okayama et al.'s research. Furthermore, compared with normal tissues (*n* = 6, Figure 1(c)), we have found that PTGR1 is observably upregulated in Garber et al.'s study that analyzed three different NSCLC histological subtypes: large cell lung carcinoma (LCC, *n* = 4, *p* = 0.017), ADC (*n* = 42, *p* = 1.17*E* − 4), and squamous cell lung carcinoma (SCC, *n* = 16, *p* = 3.56*E* − 5). Similarly, in Hou et al.'s study, PTGR1 gene is dramatically overexpressed in LCC (*n* = 19, *p* = 3.96*E* − 4), ADC (*n* = 45, *p* = 2.05*E* − 4), and SCC (*n* = 27, *p* = 7.34*E* − 7) when compared to normal lung tissues (*n* = 65, Figure 1(d)).

To confirm the above findings, we carried out qRT-PCR analysis to compare the expression of PTGR1 in human lung cancer tissues and adjacent tissues. As shown in Supplementary Figure 1, in Supplementary Material available online at http://dx.doi.org/10.1155/2016/5230642, PTGR1 was significantly increased in tumor tissues (*n* = 10, *p* = 0.0346) compared with the paired adjacent tissues (*n* = 10), which showed that consistent overexpression of PTGR1 in NSCLC tumors indicated that PTGR1 played a potential role in the carcinogenesis of the lung.

### 3.2. shPTGR1 Strongly Suppressed PTGR1 Expression in 95D and A549 Cells

To investigate the role of PTGR1 in NSCLC, lentivirus vector encoding PTGR1 shRNA was constructed and infected 95D and A549 cell lines. More than 80% of the positive GFP-expressing cells were detected under fluorescence microscopy after infection (96 h) (Figure 2(a)). To verify that the PTGR1 gene was silenced by the lentivirus vector, the mRNA and protein levels of PTGR1 expression in 95D and A549 cells were assessed using real-time quantitative PCR and western blot assays, respectively. Compared with the levels in scrambled control (shCon) cells, the knockdown efficacy of PTGR1 mRNA was 82% in 95D cells and 62.5% in A549 cells infected with shPTGR1 separately (Figure 2(b)). In addition, the expression of PTGR1 protein in 95D and A549 cells was strongly reduced (Figure 2(c)). These results indicated that shPTGR1 exerted successful knockdown effects on PTGR1 expression in 95D and A549 cells.

RETRACTED

### 3.3. shPTGR1 Suppressed the Viability and Proliferation of 95D and A549 Cells

To assess the inhibitory effect of silencing PTGR1 on cell proliferation, 95D and A549 cells were seeded on 96-well plates for a continuous 5-day MTT assay. shPTGR1 exhibited dramatic inhibition of proliferation in 95D and A549 cells compared to shCon (Figure 3(a)). The suppression of proliferation by shPTGR1 was more significant on the fifth day (*p* < 0.001). A colony formation assay was done to test whether shPTGR1 affected clonogenic potential, which is an important characteristic of tumor growth* in vivo*. As shown, silencing PTGR1 resulted in smaller clone size (Figure 3(b)) and fewer colony numbers (Figure 3(c)) compared to shCon in both 95D and A549 cells (*p* < 0.001). Taken together, the results revealed that specific PTGR1 silencing inhibits the capacity of proliferation of 95D and A549 cells.

### 3.4. shPTGR1 Arrested Cell Cycle Progression of 95D Cells

To identify the mechanism for the antiproliferation effect, cell cycle distribution was analyzed by flow cytometry after infection with shPTGR1 (Figure 4(a)). In FACS analysis in Figure 4(b), the proportion of cells in the S phase was markedly decreased (25.32%  ±  0.16% versus 32.43%  ±  0.53%, *p* < 0.001) and in G2/M-phase was increased (24.22%  ±  0.17% versus 19.09%  ±  0.57%, *p* < 0.01) in the shPTGR1 group compared with the shCon group, which represented the inhibition of cell proliferation and division. Moreover, infection of shPTGR1 into 95D cells resulted in a remarkable increase in the sub-G1 phase (0.45%  ±  0.08% versus 0.16%  ±  0.04%, *p* < 0.05, Figure 4(c)), suggesting that knockdown of PTGR1 could induce cell apoptosis.

### 3.5. shPTGR1 Promoted Cell Apoptosis in 95D Cells

In addition, we analyzed whether knockdown of PTGR1 could result in apoptosis in 95D cells. As expected, downregulation of PTGR1 induced apoptosis of 95D cells (Figures 5(a) and 5(b)). Concretely, after lentivirus transfection, the total of early and late apoptotic cells in 95D cells was 23.13% for shPTGR1, which is significantly higher than that of shCon group (10.33%, *p* < 0.001). Therefore, the ratio of apoptosis cells has significantly increased as PTGR1 was knocked down in 95D cells.

RETRACTED

### 3.6. shPTGR1 Altered the Expression of Cell Cycle Regulatory Proteins in 95D Cells

To further study the function of PTGR1 in cell cycle, the levels of cell cycle regulatory proteins were analyzed by western blot analysis. As shown in Figure 6(a), the expression of cell cycle regulatory proteins CDK2 (cyclin-dependent kinase 2), cyclin A2, CDK1 (cyclin-dependent kinase 1), and cyclin B1 was prominently reduced in shPTGR1 infected 95D cells compared with shCon infected cells. Subsequently, we further illustrated the correlation between PTGR1 and cell cycle regulatory proteins by using data mining of the Hou Lung dataset. The number of samples for each group is 45. As shown in Figure 6(b), we demonstrated that PTGR1 was positively correlated with CDK2 (*r* ^2^ = 0.12, *p* = 0.02), cyclin A2 (*r* ^2^ = 0.28, *p* < 0.001), CDK1 (*r* ^2^ = 0.11, *p* = 0.03), and cyclin B1 (*r* ^2^ = 0.19, *p* = 0.003), suggesting a possible mechanism of how PTGR1 affected the development and progress of NSCLC.

## 4. Discussion

The occurrence and development of NSCLC are closely related to the pathological state of chronic inflammation. Chen et al. reported that LTB4 may play an important role in carcinogenesis by the inflammation-augmenting and growth-stimulatory effect on tumor microenvironment and cancer cells [21]. It has been reported that LTB4 stimulated the cell proliferation in many cancers through binding with their corresponding receptors [22, 23] and was also involved in tumor angiogenesis [24]. In lung cancer, the expression of LTB4 was found to increase with progression of tumor [25] and modulated lung fibroblast functions [26]. Interestingly, PTGR1 was a key enzyme in the regulation of inflammatory mediator LTB4 [27, 28], but the biological function of PTGR1 remains largely unknown.

In the current research, a higher level of PTGR1 was expressed in NSCLC than in the normal lung tissues by using data mining of four separate lung cancer microarray datasets (Beer Lung, Okayama Lung, Garber Lung, and Hou Lung) in the Oncomine database and qRT-PCR assay. Consistent with our findings, it has also been reported that PTGR1 is significantly overexpressed in prostate cancer [29], human male germ cell tumor [30], and lymphoma [31], suggesting a potential role of PTGR1 in the carcinogenesis or malignant transformation of tumors. In further functional assays, we demonstrated that depletion of endogenous PTGR1 in 95D and A549 lung carcinoma cells inhibited cell growth, arrested cell cycle progression, and induced cell apoptosis. The above data was in a certain part in contrast with the findings reported by Zhao et al., describing PTGR1 as a tumor suppressor [32]. However, unfortunately, they did not research the expression of PTGR1 in clinical specimens. What is more, previous report has demonstrated that knockdown of PTGR1 could inhibit the growth of gastric carcinoma cells [33]. In addition, the expression level of PTGR1 was increased during hepatocellular carcinoma development [9] and also overexpression of PTGR1 decreased the survival time in bladder cancer [10]. However, some reports thought PTGR1 may be considered as a tumor suppressor because of its antioxidative and anti-inflammatory enzymatic characteristics and could enhance the efficacy of clinical antitumor chemotherapeutic drug [34–36]. We believe an important aspect to understand the role of PTGR1 in tumors is that the occurrence and development of tumor are a complex process. And, more importantly, large populations based on the analysis of Oncomine data mining have given a more objective view about how PTGR1 affects lung cancer.

RETRACTED

Certain genes may convert between oncogene and tumor suppressor under certain circumstances, such as TGF-*β* and p38. According to the literatures, TGF-*β* could suppress tumor cell growth via inducing the synthesis of 4EBP1 [37] and cyclin-dependent kinase (CDK) inhibitors such as p15, p21, and p57 [38, 39] and promote tumor cell diffusion by the induction of epithelial-mesenchymal transition (EMT) to make tumor cells get more invasion and easy to form metastases [40]. Similarly, p38 also could regulate a variety of cellular responses. It has been reported that p38 was involved in tumor cell proliferation and tumorigenesis [41, 42] and, conversely, also could negatively regulate tumor cell proliferation [43, 44]. Consequently, PTGR1 might be not just an oncogene or a tumor suppressor and the role might be altered at some stage of the oncogenesis. In addition, some studies have shown that another isoform of PTGR (PTGR2) may play a role in the occurrence and development of human tumor. Chang et al. have reported that depletion of PTGR2 inhibited the proliferation rate and induced cell apoptosis of human pancreatic cancer and gastric cancer, and PTGR2 expression is highly related to pancreatic and gastric cancers [45, 46].

To elucidate the potential regulatory mechanism of PTGR1 in tumor cell growth, we further detected alterations of some cell cycle regulators and found that there was a positive correlation between PTGR1 and cyclin-dependent proteins. CDK2/cyclin A2 protein kinase complex acts at the G1-S transition to promote the E2F transcriptional program and the initiation of DNA synthesis [47–49]. CDK1/cyclin B1 protein kinase complex plays a key role in promoting G2-M transition via association with multiple interphase cyclins [49–51]. Misregulation of CDKs can induce unscheduled proliferation and genomic and chromosomal instability [52]. As expected, it is reasonable to speculate that the mechanisms of PTGR1 knockdown suppressing the growth of lung cancer cells may be via suppression of the related cell cycle regulators to some extent.

RETRACTED

## 5. Conclusion

Our present analysis indicates the role of PTGR1 in lung cancer. The above data suggested that PTGR1 mediated lung cell survival through cell cycle arrest and apoptosis. PTGR1 promoted lung cancer growth by regulating the expression of intracellular related cell cycle protein, but the exact mechanism needs further analysis. Therefore, PTGR1 gene may be considered as a novel candidate target for lung cancer.

## Supplementary Material

Supplementary Figure 1: Expression of PTGR1 in lung cancer tissues and corresponding normal tissues. qRT-PCR was performed to evaluate the PTGR1 mRNA expression in lung cancer tissues and adjacent normal lung tissues (*n*=10, *p*<0.05).

## Figures and Tables

**Figure 1:** Overexpression of PTGR1 mRNA in NSCLC was revealed by data mining of the Oncomine database. (a) The expression of PTGR1 was upregulated in ADC tissues compared with the normal lung tissues revealed using the Beer Lung database. (b) Differential expression of PTGR1 in the normal and ADC tissues was revealed by the Okayama Lung dataset. (c) PTGR1 expression analysis in the lung, LCC, ADC, and SCC tissues in the Garber Lung dataset was shown. (d) PTGR1 expression in the lung, LCC, ADC, and SCC specimens in the Hou Lung dataset was different. The total number of samples was shown under each category. The *p* values were calculated using two-tailed and unpaired Student's *t*-test.

**Figure 2:** Silencing of PTGR1 in 95D and A549 cells by shPTGR1-expressing lentivirus. (a) Images of 95D and A549 cells 72 h after shPTGR1 infection under inverted fluorescent microscope with the magnification of 100x. (b) Real-time PCR analysis. PTGR1 mRNA in 95D/shPTGR1 and A549/shPTGR1 was decreased significantly when compared to 95D/shCon and A549/shCon cells. Values were expressed as mean ± SD. (c) Western blotting analysis. PTGR1 protein in 95D/shPTGR1 and A549/shPTGR1 was decreased significantly compared to 95D/shCon and A549/shCon cells. ^*∗∗*^ *p* < 0.01; ^*∗∗∗*^ *p* < 0.001.

**Figure 3:** shPTGR1 inhibited the proliferation of 95D and A549 cells. (a) The growth curve in 95D/shPTGR1 and A549/shPTGR1 was lower than in 95D/shCon and A549/shCon cells. (b) Images recorded under micro and macro view, representing the size and the number of colonies in each group of cells. All data represented as mean value ± SD from 3 independent experiments. (c) Statistical analysis revealed that the number of colonies in 95D/shPTGR1 and A549/shPTGR1 was lower than in 95D/shCon and A549/shCon cells. ^*∗∗*^ *p* < 0.01; ^*∗∗∗*^ *p* < 0.001.

RETRACTED

**Figure 4:** shPTGR1 inhibited the cell cycle progress of 95D cells. (a) FACS analyses of cell cycle distribution in 95D cells. A hypodiploid apex representing the apoptotic cells was found before the G1 apex in 95D/shPTGR1. (b) Downregulation of PTGR1 in 95D cells led to an increase of cells at G2/M phase and concomitantly a decrease of cells at S phase. (c) Downregulation of PTGR1 in 95D cells led to an increase of cells at sub-G1 phase. Data represents means ± SD from 3 independent experiments. ^*∗*^ *p* < 0.05; ^*∗∗*^ *p* < 0.01; ^*∗∗∗*^ *p* < 0.001.

**Figure 5:** shPTGR1 induced 95D cell apoptosis. (a) In shCon and shPTGR1 groups, the representative FACS analysis is as shown. (b) The proportion of early and late apoptosis was revealed. Data are reported as means ± SD of three independent experiments. ^*∗∗∗*^ *p* < 0.001, compared to shCon.

**Figure 6:** shPTGR1 affected the expression of cell cycle regulatory proteins. (a) The levels of CDK1, cyclin A2, CDK2, and cyclin B1 protein were analyzed by western blot in shCon and shPTGR1 infected 95D cells. GAPDH was used as an internal loading control. (b) Correlation between PTGR1 and CDK1/cyclin A2/CDK2/cyclin B1 mRNA expression in lung cancer is observed. Pearson's correlation coefficient test.
